The article "Length of Stay Prediction Model of Indoor Patients Based on Light Gradient Boosting Machine" was published in 2022. Journal: Comput Intell Neurosci.

# Length of Stay Prediction Model of Indoor Patients Based on Light Gradient Boosting Machine

**DOI:** 10.1155/2022/9517029

**Published:** 2022-08-30

**Authors:** Xiangrui Zeng

**Affiliations:** School of Computer Sciences, Universiti Sains Malaysia, Penang 11800, Malaysia

## Abstract

The influx of hospital patients has become common in recent years. Hospital management departments need to redeploy healthcare resources to meet the massive medical needs of patients. In this process, the hospital length of stay (LOS) of different patients is a crucial reference to the management department. Therefore, building a model to predict LOS is of great significance. Five machine learning (ML) algorithms named Lasso regression (LR), ridge regression (RR), random forest regression (RFR), light gradient boosting machine (LightGBM), and extreme gradient boosting regression (XGBR) and six feature encoding methods named label encoding, count encoding, one-hot encoding, target encoding, leave-one-out encoding, and the proposed encoding method are used to construct the regression prediction model. The Scikit-Learn toolbox on the Python platform builds the prediction model. The input is the dataset named Hospital Inpatient Discharges (SPARCS De-Identified) 2017 with 2343569 instances provided by the New York State Department of Health verify the model after removing 2.2% of the missing data, and the model ultimately uses mean squared error (MSE) and coefficient of determination (*R*^2^) as the performance measurement. The results show that the model with the LightGBM algorithm and the proposed encoding method has the best *R*^2^ (96.0%) and MSE score (2.231).

## 1. Introduction

Globally, due to the pandemic and population changes, hospital inpatient departments are becoming more and more likely to face the influx and congestion of patients [1, 2] and hospitals in anticipation of the need to redeploy healthcare resources to meet the massive medical requirements of patients [3]. The LOS indicates the number of days between admission and discharge, and it can often affect the admission plan of emergency patients [4] or whether there is the possibility of transfer [5]. Moreover, when technical means can reduce the long duration of LOS, the consumption of healthcare resources would also be reduced to some extent [6]. However, the inpatient department does not know when existing patients will leave the hospital in most cases. If hospitals could accurately predict LOS, they could implement and improve healthcare resource management correctly [7, 8]. Therefore, this study tries to establish an ML model using the information about the diagnosis, treatment, service, and cost of individual patients to predict LOS.

The article "Length of Stay Prediction Model of Indoor Patients Based on Light Gradient Boosting Machine" was published in 2022. Journal: Comput Intell Neurosci.

In the study, five ML algorithms (LR, RR, RFR, XGBR, and LightGBM) and six feature encoding methods (label encoding, count encoding, one-hot encoding, target encoding, leave-one-out encoding, and the proposed encoding method) were used and compared during the model building. The rest of the study is organized as follows: Section 2 reviews some related studies on LOS.  Section 3 introduces the dataset used in this study and each step of the proposed framework in detail.  Section 4 presents the experimental results and then discusses them.  Section 5 draws the conclusions and direction of future work.

## 2. Related Works

Several researchers have conducted related studies on predicting hospital LOS. Some of them discrete the LOS value that transforms the regression problem into classification. For example, Bacchi et al. [9] proposed an artificial neural network (ANN)-based prediction model for predicting the LOS in stroke patients. The objective is to predict whether the LOS was less than 8 days. And they finally achieved 0.62 and 0.66 area under curve (AUC) values on the inner and outer validation sets. Similarly, Daghistani et al. [10] converted the LOS values into three classes (<3 days, 3–5 days, and >5 days) and then used information gain (IG) to select features. They compared Random Forest (RF), Bayesian Network (BN), Support Vector Machine (SVM), and ANN technology for LOS prediction. The final RF model outperformed all other models (sensitivity (0.80), accuracy (0.80), and AUROC (0.94)). Furthermore, Zheng et al. [11] compared two discrete methods that are two (1-3 days and ≥4 days) and three (1–3 days, 4-8 days, and ≥9 days) classes. Six ML algorithms were applied to the model to make comparative predictions and finally obtained the best accuracy score (ACC) of 0.7689 and 0.6594 in the training and test sets, respectively. Furthermore, Ling et al. [12] used the RF algorithm and general medical characteristics to predict LOS in patients in the intensive care unit (ICU), and the AUC value of the optimal model is 0.86.

The limitation of classification-type studies is their generally poor performance and difficulty in guiding long-term LOS (e.g., LOS ≥ 10 days) prediction due to the small number of classes. Models of this discrete type are unrealistic to deploy and not recommended when hospitals hope to predict the LOS precisely (e.g., ±1 day).

Data balancing techniques can improve model performance in predicting LOS. For example, Naemi et al. [13] proposed a multistage data processing method. The method first used k-nearest neighbors (KNN), decision tree (DT), gradient boosting (GB), Bayesian ridge (BR), Gaussian process (GP), and RF for missing value imputation and then used SMOTE to overcome data skewness. After these steps, the model used DT to predict the hours of stay. It ended up with an *R*^2^ score of 0.729. Alsinglawi et al. [14] constructed a LOS prediction framework for lung cancer patients using RF and oversampling techniques (SMOTE and ADASYN). The framework gets an AUC score of 100% on the MIMIC-III dataset.

The article "Length of Stay Prediction Model of Indoor Patients Based on Light Gradient Boosting Machine" was published in 2022. Journal: Comput Intell Neurosci.

The datasets used in the above two studies have been artificially altered. Even though model performance is good on synthetic balanced data, it often does not perform well on unbalanced data. As a result, models using data balancing techniques are difficult to deploy because data tend to be biased in real life.

According to historical data, regression is the method that occupies the majority proportion of LOS prediction [15]. For example, Siddiqa et al. [16] used multiple linear regression (MLR), decision tree regression (DTR), LR, RR, XGBR, and RFR techniques to predict LOS. They found that RFR is the best model that achieved the 5 MSE and 0.92 *R*^2^ scores. In another study, Abbas et al. [17] established a model based on multilayer perceptron (MLP) to predict LOS for total knee arthroplasty. The model uses medical data such as a patient's white blood cell count and type of anesthesia, and finally received 0.715 and 0.690 MSE scores on training and test sets, respectively. Zhong et al. [18] compared three models based on backpropagation neural network (BPNN), support vector regression (SVR), and principal component regression (PCR). The best experimental result of the 1.5254 mean absolute error (MAE) score is on the PCR model. The study of Kolchun et al. [19] established a prediction model for passenger LOS after a motor vehicle collision. After comparing various ML methods, the MAE of LOS prediction by the neural network (NN) algorithm reaches 2.23.

Previous regression models have two limitations. First, some models are built on specific or posthospital physical examination data, so they lack generality. The other model built on datasets with high versatility is insufficient in performance (*R*^2^ < 0.95). Based on the deficiencies of the three model types, this study attempts to propose a model that does not use artificially synthesized data and excels in both generality (e.g., using prehospital diagnosis results) and performance.

## 3. Materials and Methods

### 3.1. Data Description

The study used the Hospital Inpatient Discharges (SPARCS De-Identified) 2017 dataset provided by the New York State Department of Health [20]. This dataset uses the Open Database License (ODbL 1.0), which grants anyone to use the dataset for the duration of any applicable copyright and Database Rights. These rights explicitly include commercial use and do not exclude any field of endeavor [21]. The dataset contains 2343569 instances with 34 features that de-identify the detailed information of patient characteristics, diagnosis, treatment, services, and costs. The “Length of Stay” in the dataset is the target feature, while the purpose of the proposed model is to predict it by others.  Table 1 shows the description of the features of the dataset.

The article "Length of Stay Prediction Model of Indoor Patients Based on Light Gradient Boosting Machine" was published in 2022. Journal: Comput Intell Neurosci.

### 3.2. The Proposed Framework

This study uses a few steps to build a complete application model. First, the raw data use visualization to analyze the internal relationship, and then the data are preprocessed for duplicates, missingness, and meaningless information. The third step determines whether each feature of the dataset positively affects the target, and the model only needs the positive partial. Then the six encodings make the information in the dataset unusable into a usable form.

The above steps make modifications to the raw data. Then the model divides data into a training set and a test set in a 99: 1 ratio, where the training set uses a 10-fold cross-validation technique to improve model reliability. After the five ML algorithms have trained the model, MSE and *R*^2^ will judge the model performance to support analysis.

Figure 1 presents the framework proposed in this study. And this framework fully expresses the methodology used to construct the model for this study. The following sections explain each step of the framework in detail.

### 3.3. Data Visualization Analysis

The study leverages visualization techniques to analyze datasets and find relationships between independent and dependent features. The results produced by visualization methods are usually easily understandable by people who are not necessarily knowledgeable about ML [22].  Table 1 shows that the dataset has two or three class categorical, ordered categorical, random categorical, and continuous features, in which the target “Length of Stay” belongs to the continual type.

Figure 2 shows the density distribution of the target feature. It belongs to the long-tail distribution with an average value of 5.38. Therefore, all analysis methods that assume the normal distribution are less suitable for this study.  Figure 3 shows the proportion of LOS in different categories of patients in the three features of “Gender,” “APR Medical Surgical Description,” and “Emergency Department Indicator.” The results showed that the LOS of the female patients was longer than that of the male patients but was uniform. In the middle of the figure, the LOS of medical inpatients accounts for about three-quarters of the total, of which the type is much longer than surgical inpatients. And the LOS of emergency patients is about twice that of nonemergency patients, showing that the condition of emergency patients is more ill and needs a longer recovery time.  Figure 4 shows the density distribution of two continuous features, and the trend is similar to Figure 2. This figure demonstrates that the two features correlate with the target. Finally, Figure 5 shows the LOS of two ordered categorical features, which shows that the younger the age and the higher the disease mortality rate, the shorter the LOS.

The article "Length of Stay Prediction Model of Indoor Patients Based on Light Gradient Boosting Machine" was published in 2022. Journal: Comput Intell Neurosci.

### 3.4. Data Preprocessing

Outliers and missing values during model building would affect the model performance [23], then data preprocessing is crucial. Among the 34 features, the missing value of “Payment Type 2” is missing completely at random (MCAR) and is missing at random (MAR) [24] in “Payment Typology 3” and “Birth Weight.” The proportion of their missing values is about 37.5%, 74.1%, and 90.3% [25]. Hence the process removed three features directly. The remaining dataset also needs to remove about 2% of the instances that still contain MCAR or MAR, as well as 20 samples with the value of “Unknown” in the “Gender” feature. It is worth mentioning that all eigenvalues “120+” were uniformly changed to “120” for the convenience of calculation in the feature “Length of Stay.” Finally, there are 2304296 instances with 31 features left in the dataset that the preprocessing process deleted 2.2% instances.

### 3.5. Feature Selection

Among the remaining 31 features of the dataset after preprocessing, the five features of “CCS Diagnosis Description,” “CCS Procedure Description,” “APR DRG Description,” “APR MDC Description,” and “APR Severity of Illness Description” are different representations of the same information as the five features of “CCS Diagnosis Code,” “CCS Procedure Code,” “APR DRG Code,” “APR MDC Code,” and “APR Severity of Illness Code,” respectively, which are meaningless to the model and therefore deleted.

Among the 24 remaining features of the dataset, the “Length of Stay” is the continuous target feature. And others are divided into four types (Binary, Ordered Categorical, Random Categorical, and Continuous). Regarding the correlation between them and the target feature, it is necessary to use various techniques to investigate.

#### 3.5.1. Binary Features

The point-biserial correlation is the value of Pearson's product-moment correlation when one of the variables is dichotomous and the other variable is metric [26]. The calculation formula of the point-biserial correlation coefficient is as follows:

(1) $$\begin{array}{c} \gamma_{pb}=\frac{\bar{Y_{1}}-\bar{Y_{0}}}{\bar{s_{n}}}\sqrt{\frac{n_{1}n_{0}}{n\left(n-1\right)}}, \end{array}$$

where *n*_1_ and $\bar{Y_{1}}$ represent the frequency of the binary feature *X*=1 and the mean of the corresponding target feature, respectively. *n*_0_ and $\bar{Y_{0}}$ represent the frequency of the binary variable *X*=0 and the mean of the corresponding target feature, respectively. And the $\bar{s_{n}}$ in the denominator represents the standard deviation of the target feature [26]. Finally, the closer the absolute value of *γ*_*pb*_ is to 1, the higher the correlation between features.

The article "Length of Stay Prediction Model of Indoor Patients Based on Light Gradient Boosting Machine" was published in 2022. Journal: Comput Intell Neurosci.

#### 3.5.2. Ordered Categorical Features

The correlation of ordered categorical features with continuous features requires first converting the latter to the former type. The two most popular measures of association for this feature type are Kendall's tau and Spearman's rho [27]. This study uses the Spearman coefficient for correlation analysis, and the general idea is as follows:

The method of Spearman first converts the string data *X*^*i*^=[*X*_1_^*i*^, *X*_2_^*i*^,…*X*_*n*_^*i*^] in the ordered categorical features into numerical grade data *x*^*i*^=[*x*_1_^*i*^, *x*_2_^*i*^,…*x*_*n*_^*i*^].  Table 2 shows the conversion detail. And the data *y*=[*y*_1_=1, *y*_2_=2,…*y*_*n*_=120] in the target feature are used directly without modification. The method then uses formula (2) [28, 29] to calculate the correlation between *x* and *y*. The absolute value of the result *ρ*_*X*,*Y*_ is between 0 and 1, and the closer to 1, the more correlated the features are.

(2) $$\begin{array}{c} \rho_{x,y}=\frac{\sum \left(x-\bar{x}\right)\left(y-\bar{y}\right)}{\sqrt{\sum {\left(x-\bar{x}\right)}^{2}}\sqrt{\sum {\left(y-\bar{y}\right)}^{2}}}. \end{array}$$

#### 3.5.3. Random Categorical Features

Since the target feature does not satisfy the normal distribution (Figure 2), it is suitable to use the Kruskal–Wallis test to calculate the correlation with the target feature. The Kruskal–Wallis test is a nonparametric statistical test that assesses the differences among three or more independently sampled groups on a single, nonnormally distributed continuous feature [30]. The basic idea is as follows:

The Kruskal–Wallis test first arranges the eigenvalues in ascending order, then finds their rank *R*_*i*_, and examines whether there is a significant difference in the mean *μ*_*i*_ of the ranks of each eigenvalue. *H*_0_ : *μ*_1_ = *μ*_2_ = …*μ*_*k*_ is the null hypothesis, and the alternative hypothesis H1 is that at least two *μ*_*i*_ are not equal. The calculation formula [31] is as follows:

(3) $$\begin{array}{c} H=\frac{12}{N\left(N+1\right)}\overset{\underset{k}{i=1}}{\Sigma }n_{i}{\bar{R}}_{i}^{2}-3\left(N+1\right). \end{array}$$

Through *H* in the above formula, the Kruskal–Wallis test can query the critical value table to get the corresponding *P* value. If the *P* value is below the significance level, there is a correlation between the features. And this study sets the threshold at 0.01.

The article "Length of Stay Prediction Model of Indoor Patients Based on Light Gradient Boosting Machine" was published in 2022. Journal: Comput Intell Neurosci.

#### 3.5.4. Continuous Features

Since the target feature is not normally distributed (Figure 2), its correlation with continuous features needs to be judged by the Spearman correlation coefficient [32].

Finally, Table 3 summarizes the correlation between each feature and the target feature. And the results show the model could keep all features.

### 3.6. Feature Encoding

All categorical attributes of the dataset are represented by strings, while machine learning algorithms can only calculate numerical eigenvalues. Hence these features need to be rerecorded into numbers.

#### 3.6.1. Label Encoding

In the label encoding method, the eigenvalues of each categorical feature are first sorted by frequency from small to large and then are assigned a value from 0 to N−1 in order (N indicates how many different eigenvalues the feature has). Even if there is no relationship between the eigenvalues before encoded, the algorithm would regard them according to the size of the values.  Table 4 shows a sample of this method on one particular feature.

#### 3.6.2. Count Encoding

Count encoding is a method that uses the frequency of eigenvalues as labels. In this method, the frequency of one feature will replace the value of this feature. And different eigenvalues may be encoded into the same number. When the frequency of categorical features correlates with the target feature, this method has positive significance for model training.

#### 3.6.3. One-Hot Encoding

When a feature with *M* unique values, one-hot encoding will create *M* corresponding new features, where the new value (1 or 0) indicates whether the instance has the represented original categorical value.  Table 5 demonstrates the principle of one-hot encoding. However, there are too many eigenvalues in discrete features in the dataset. If all features use one-hot encoding, more than 1500 new will be generated and will be too sparse. Hence, only features with a small number of unique values will use this method.

#### 3.6.4. Target Encoding

Target encoding is a preprocessing scheme for high-cardinality categorical features based on a well-established statistical approach to models (empirical Bayes). It is a method based not only on the independent eigenvalues but also on the corresponding dependent feature [33]. This method depends on the distribution of dependent features, but the feature dimension remains unchanged after encoding, and its calculation formulas (4) and (5) [33] are as follows:

(4) $$\begin{array}{c} S_{i}=\lambda \left(n_{i}\right)\frac{\sum_{k\in L_{i}}Y_{k}}{n_{i}}+\left(1-\lambda \left(n_{i}\right)\right)\frac{\sum_{k=1}^{N_{TR}}Y_{k}}{n_{TR}}, \end{array}$$

(5) $$\begin{array}{c} \lambda \left(n_{i}\right)=\frac{1}{1+e^{-\left(n-k/f\right)}}. \end{array}$$

In formula (4), ∑_*k*∈*L*_*i*__*Y*_*k*_ represents the sum of the corresponding target feature's values when the categorical eigenvalue is *i*. Its denominator *n*_*i*_ represents the frequency of categorical eigenvalue *i*. And the ∑_*k*=1_^*N*_*TR*_^*Y*_*k*_ on the right side of the formula represents the sum of the values of the target feature in the training set.

*k* in formula (5) represents the minimum times the eigenvalue must appear in the calculated feature. And *λ* represents the smoothing coefficient that the higher the value, the stronger the regularization of the formula.

The article "Length of Stay Prediction Model of Indoor Patients Based on Light Gradient Boosting Machine" was published in 2022. Journal: Comput Intell Neurosci.

#### 3.6.5. Leave-One-Out Encoding

The leave-one-out encoding method uses the same principle and formula as target encoding. But to reduce the influence of outliers, when calculating the encoding value of an instance, the program will ignore the current and only use the remaining for target encoding.

#### 3.6.6. Proposed Encoding Method

One-hot encoding method can obtain the information of categorical features well, but it will lead to sparse data. The other methods do not have the problem of sparsity but will lose a lot of data information. This study attempts to balance model performance and data dimensionality, thus combining two encodings to form a new method.  Table 6 shows the encoding adopted for each feature.

### 3.7. Comparative Algorithms

#### 3.7.1. Lasso Regression

LR is to fit the dataset *D*={(*x*_1_^1^, *x*_1_^2^,…, *x*_1_^*m*^, *y*_1_), (*x*_2_^1^, *x*_2_^2^,…, *x*_2_^*m*^, *y*_1_),…, (*x*_*n*_^1^, *x*_*n*_^2^,…, *x*_*n*_^*m*^, *y*_1_)} (*m* represents the number of features and *n* indicates the number of instances) with a linear function (6) and minimize the cost function (7) [34], where *f*(*x*) represents the predicted values and *y*_*i*_ is true values. The purpose of the operation is to find a solution (*W*, *b*) that minimizes *J*(*w*). LR imposes constraints on the model parameters (i.e., adds a penalty *λ*‖*w*_*j*_‖ to the loss function) that shrink the regression coefficients to zero [35]. For example, if a feature highly correlates with the target, LR will select it and then shrink others uncorrelated with zero and exclude them from the model. This approach reduces bias and improves the accuracy of linear regression models.

(6) $$\begin{array}{c} f\left(x\right)=W^{T}\cdot X+b \end{array}$$

(7) $$\begin{array}{c} J\left(w\right)=\sum_{i=1}^{m}{\left(y_{i}-\sum_{j=0}^{n}w_{j}x_{j}^{\left(i\right)}\right)}^{2}+\lambda \left\|w_{j}\right\|. \end{array}$$

By calculating the partial derivative concerning *w* of the residual on the left side and the penalty term on the right side of formula (7) could obtain formulas (8) and (9).

(8) $$\begin{array}{c} \frac{\partial }{\partial w_{k}}RSS\left(w\right)=-2\sum_{i=1}^{m}\left(x_{k}^{\left(i\right)}y^{\left(i\right)}-x_{k}^{\left(i\right)}\sum_{j=0,j\neq k}^{n}w_{j}x_{j}^{\left(i\right)}-w_{k}x_{k}^{{\left(i\right)}^{2}}\right), \end{array}$$

(9) $$\begin{array}{c} \frac{\partial }{\partial w_{k}}R\left(w\right)=\left\{\begin{array}{cc} -\lambda , & w_{k}<0,\\ \left[-\lambda ,\lambda \right], & w_{k}=0,\\ \lambda , & w_{k}>0, \end{array}\right. \end{array}$$

where *x*_*k*_^(*i*)^∑_*j*=0,*j*≠*k*_^*n*^*w*_*j*_*x*_*j*_^(*i*)^ − *w*_*k*_*x*_*k*_^(*i*)^2^^=*x*_*k*_^(*i*)^∑_*j*=0_^*n*^*w*_*j*_*x*_*j*_^(*i*)^. Set *P*_*k*_=∑_*i*=1_^*m*^[*x*_*k*_^(*i*)^(*y*^(*i*)^ − ∑_*j*=0,*j*≠*k*_^*n*^*w*_*j*_*x*_*j*_^(*i*)^)] and *Z*_*k*_=∑_*i*=1_^*m*^*x*_*k*_^(*i*)^2^^, then combine (8) and (9) to obtain the partial derivative of (7) and solve it:

(10) $$\begin{array}{c} w_{j}=\left\{\begin{array}{cc} \frac{\left(P_{k}+\left(\lambda /2\right)\right)}{Z_{k}}, & P_{k}<-\left(\frac{\lambda }{2}\right),\\ 0, & -\left(\frac{\lambda }{2}\right)\leq P_{k}\leq \left(\frac{\lambda }{2}\right),\\ \frac{\left(P_{k}-\left(\lambda /2\right)\right)}{Z_{k}}, & P_{k}>\left(\frac{\lambda }{2}\right). \end{array}\right. \end{array}$$

The article "Length of Stay Prediction Model of Indoor Patients Based on Light Gradient Boosting Machine" was published in 2022. Journal: Comput Intell Neurosci.

#### 3.7.2. Ridge Regression

RR is similar to LR and uses the linear formula (6). It obtains regression coefficients at the cost of losing some information and reducing accuracy by giving up unbiasedness. RR adds a penalty term to the loss function in standard linear regression to alleviate multicollinearity and overfitting problems [36]. Its estimates of regression coefficients tend to become too large in absolute values, and some may even have the wrong sign [37]. Formula (11) [38] is the loss function of RR, which is the penalty term added by *λ*‖*w*_*j*_‖^2^. And *λ* is a hyper-parameter used to control the strength of the penalty. The larger the *λ*, the simpler the generated model.

(11) $$\begin{array}{c} J_{\beta }\left(\beta \right)=\overset{n}{\underset{i=1}{\sum }}{\left(y_{i}-\underset{j}{\sum }w_{j}x_{j}^{\left(i\right)}\right)}^{2}+\lambda {\left\|w_{j}\right\|}^{2}. \end{array}$$

#### 3.7.3. Random Forest Regression

RFR adopts the Bootstrap [39] technique to randomly divide the dataset *D* into *n* subsample sets {*D*_1_, *D*_2_,…, *D*_*n*_}. The CART regression tree will build on these subsets and output the results, and the final RFR outputs the average of all predictions. There is no relationship between each regression tree, an increase in the number of trees does not cause the RFR to overfit the data [40]. Furthermore, RFR is insensitive to multicollinearity, and the results are robust to missing and unbalanced data [41].

The article "Length of Stay Prediction Model of Indoor Patients Based on Light Gradient Boosting Machine" was published in 2022. Journal: Comput Intell Neurosci.

The 31 features of each divided subsample set *D*_*i*_ are set to *A*={*A*_1_, *A*_2_,…, *A*_31_}. The CART algorithm first sorts the features *A*_*i*_ and then tries to use each interval between adjacent feature values as the segmentation point *S*. The set of eigenvalues on the left side of *S* is *R*_1_ (*A*_*i*_, *S*) and the right side is *R*_2_ (*A*_*i*_, *S*) (12). *c*_1_ and *c*_2_ are the mean values of the target feature corresponding to *R*_1_ (*A*_*i*_, *S*) and *R*_2_ (*A*_*i*_, *S*), respectively (13). The next step of the algorithm is to find which *S* can make the MSE of the feature minimum (14) and then use the segmentation point *S* together with the feature as the node of the tree. After the algorithm divides all features, the CART regression tree uses the average of all leaf nodes as the output (15) [42].

(12) $$\begin{array}{c} R_{1}\left(A_{i},S\right)=\left\{x|x^{A_{i}}\leq S\right\},\\ R_{2}\left(A_{i},S\right)=\left\{x|x^{A_{i}}\leq S\right\}, \end{array}$$

(13) $$\begin{array}{c} c_{1}=\text{ave}\left(y_{i}|x_{i}\in R_{1}\left(A_{i},S\right)\right),\\ c_{2}=\text{ave}\left(y_{i}|x_{i}\in R_{2}\left(A_{i},S\right)\right), \end{array}$$

(14) $$\begin{array}{c} \min_{A_{i},s}=\left[\min_{c_{1}}\sum_{x_{i}\in R_{1}\left(A_{i},s\right)}{\left(y_{i}-c_{1}\right)}^{2}+\min_{c_{2}}\sum_{x_{i}\in R_{2}\left(A_{i},s\right)}{\left(y_{i}-c_{2}\right)}^{2}\right], \end{array}$$

(15) $$\begin{array}{c} f\left(x\right)=\sum_{m=1}^{31}c_{m}I\left(x\in R_{m}\right). \end{array}$$

#### 3.7.4. Extreme Gradient Boosting Regression

Unlike RFR in the bagging form, XGBR is a boosting integrated ML algorithm based on the CART regression tree, which belongs to the regression implementation of extreme gradient boosting (XGBoost). It uses the second-order Taylor expansion and adds regularization to the objective function. And the algorithm adopts accurate greedy ideas in the tree generation [43]. Finally, XGBR uses the sum of the predictive values of all regression trees for the sample as the output of this sample in the system, and the definition function (16) [43] is as follows:

(16) $$\begin{array}{c} {\hat{y}}_{i}=\sum_{k=1}^{K}f_{k}\left(X_{i}\right),\;f_{k}\in F, \end{array}$$

where *X*_*i*_ is the sample feature and *f*_*k*_(*X*_*i*_) is the prediction of the *K*th tree. The sum of values of all trees is the predicted value ${\hat{y}}_{i}\;$ for the entire model. Since the algorithm belongs to the additive model, the predicted value of the *K*th tree ${\hat{y}}_{i}^{k}$ can be expressed by formula (17). Let the sum of the truth values be *y*_*i*_. Formula (18) [43] summarizes the objective function.

(17) $$\begin{array}{c} {\hat{y}}_{i}^{k}={\hat{y}}_{i}^{k-1}+f_{k}\left(X_{i}\right), \end{array}$$

(18) $$\begin{array}{c} \text{min}\left(L\left(\varphi \right)=\underset{i}{\sum }l\left({\hat{y}}_{i},y_{i}\right)+\underset{k}{\sum }\Omega \left(f_{k}\right)=\underset{i}{\sum }l\left(f_{k}\left(X_{i}\right)+{\hat{y}}_{i}^{k-1},y_{i}\right)+\underset{k}{\sum }\Omega \left(f_{k}\right)\right), \end{array}$$

where ∑_*k*_Ω(*f*_*k*_)=∑_*i*=1_^*K*−1^Ω(*f*_*j*_)+Ω(*f*_*K*_). $\sum_{i}l\left({\hat{y}}_{i},y_{i}\right)$ is the loss function between the predicted and true values that is MSE (11) in XGBR. Since the results of K-1 trees have been determined and remain unchanged when training the *K*th tree, ∑_*k*_Ω(*f*_*k*_) can convert to Ω(*f*_*K*_). Then, the Taylor expansion can transform the objective function on the right side of formula (18) into (19).

(19) $$\begin{array}{c} \text{min}\left(L\left(\varphi \right)≃\underset{i}{\sum }\left[l\left({\hat{y}}_{i}^{k-1},y_{i}\right)+g_{i}\cdot f_{k}\left(X_{i}\right)+\frac{1}{2}h_{i}\cdot f_{k}^{2}\left(X_{i}\right)\right]+\Omega \left(f_{K}\right)\right), \end{array}$$

where $\sum_{i}l\left({\hat{y}}_{i}^{k-1},y_{i}\right)$ is the sum of the prediction losses of the first *K*-1 trees. And it does not change when computing the *K*th tree and can therefore be ignored. $g_{i}=\partial_{{\hat{y}}_{i}^{\left(k-1\right)}}l\left({\hat{y}}_{i}^{k-1},y_{i}\right)$ and $h_{i}=\partial^{2}{}_{{\hat{y}}_{i}^{\left(k-1\right)}}l\left({\hat{y}}_{i}^{k-1},y_{i}\right)$ can be treated as a constant too. *f*_*k*_(*X*_*i*_) represents the prediction result of the *K*th tree, and it also indicates the leaf node position on the *K*th tree where the sample *X*_*i*_. Here, the function *q*(*X*_*i*_) can be defined to represent the sample position in leaf nodes, and *w*_*q*(*X*_*i*_)_=*f*_*k*_(*X*_*i*_) can express to solve the sample position. XGBoost defines Ω(*f*_*K*_)=*γT*+1/2*λ*∑_*t*=1_^*T*^(*ω*_*t*_)^2^ as the penalty function (where *λ* represents the penalty intensity and *T* is the number of leaf nodes) [43]. Formula (19) can convert to formula (20) by removing the constant term and substituting the penalty.

(20) $$\begin{array}{c} \text{min}\left(L\left(\varphi \right)=\underset{i}{\sum }\left[g_{i}\cdot w_{q\left(X_{i}\right)}+\frac{1}{2}h_{i}\cdot w_{q\left(X_{i}\right)}^{2}\right]+\gamma T+\frac{1}{2}\lambda \overset{T}{\underset{t=1}{\sum }}{\left(\omega_{t}\right)}^{2}=\overset{T}{\underset{j=1}{\sum }}\left[\left(\underset{i\in I_{j}}{\sum }g_{i}\right)\cdot w_{j}+\frac{1}{2}\left(\underset{i\in I_{j}}{\sum }h_{i}+\lambda \right)\cdot w_{j}^{2}\right]+\gamma T\right), \end{array}$$

where only *w*_*j*_ is unknown, so the objective function becomes a typical quadratic type. XGBR adopts the CART regression tree that could fix the tree structure *q*(*X*_*i*_). At this time, the minimum solution of the function is *w*_*j*_^*∗*^=−((∑_*i*∈*I*_*j*__*g*_*i*_)/(∑_*i*∈*I*_*j*__*h*_*i*_+*λ*)), substituting into formula (20) can get the objective function solution −(1/2)∑_*j*=1_^*T*^((∑_*i*∈*I*_*j*__*g*_*i*_)^2^/(∑_*i*∈*I*_*j*__*h*_*i*_+*λ*))+*γT*.

The article "Length of Stay Prediction Model of Indoor Patients Based on Light Gradient Boosting Machine" was published in 2022. Journal: Comput Intell Neurosci.

#### 3.7.5. Light Gradient Boosting Machine

Microsoft launched an upgraded version of XGBoost named LightGBM in 2017. The LightGBM in this article uses the histogram algorithm to reduce the number of candidates' split points and the mutually Exclusive Feature Bundling (EFB) algorithm to reduce the number of features [44].

The histogram algorithm refers to discretizing continuous floating-point eigenvalues into *k* integers and constructing a histogram with a width of *k*. The algorithm counts the floating-point values within the range of the discretized values in the histogram according to the *k* values as an index. Then traverses the discretized values to find the optimal segmentation point. XGBoost travels all floating-point values, while LightGBM only travels *k* values by establishing histograms. EFB will compare and analyze the difference between features by sparse coding. When the difference between the two features is minor, it considers that there is a conflict. Otherwise, the two features will be one. EFB reduces the feature dimension through this method to speed up.

Hence LightGBM is more efficient run on the set in large-scale data. With the same performance as XGBR, LightGBM is 10x faster than train and consumes less memory [44].

### 3.8. Model Validation

Although the dataset has more than 2 million instances, the model is still at risk of overfitting. Secondarily, the model training process is necessary to avoid information leakage caused by using the test set multiple times. Based on the above factors, the validation process divides the dataset into a training set and a test set in a 99:1 ratio. Then the training set is used for 10-fold cross-validation, and the test set checks the model performance. The entire validation process will use the training set ten times, but the test set only once.

The 10-fold cross-validation method could alleviate the overfitting and information leak [45]. The reason for choosing 10 is the estimate of prediction error is almost unbiased [46]. The 10-fold method will use different 90% training sets to train the model ten times, and the remaining measures the model performance.

The article "Length of Stay Prediction Model of Indoor Patients Based on Light Gradient Boosting Machine" was published in 2022. Journal: Comput Intell Neurosci.

### 3.9. Performance Measurement

The model in this study attempts to solve a regression problem, in which people usually achieve model performance measurement by comparing the MSE and *R*^2^. The closer the MSE value is to 0, the smaller the gap between the predicted and the actual value. Formula (21) [47] calculates the MSE by subtracting each prediction from the truth, adding all the squared results, and dividing by the total number added.

(21) $$\begin{array}{c} MSE=\frac{1}{n}\sum {\left(y_{i}-\hat{y}\right)}^{2}, \end{array}$$

where *y*_*i*_ represents the actual value, $\hat{y}$ represents the predicted value, and *n* represents the total number of squared values.

When the dimensions are different, MSE does not say much about the performance of the regression concerning the distribution of the ground truth elements. However, the *R*^2^ score does not have the interpretability limitations of MSE and is more informative and truthful [48]. The value of the *R*^2^ score is between −*∞* and 1. *R*^2^ = 1 indicates the predicted values are the same as the actual values. Hence, the closer the score is to 1, the better the model performance. Formula (22) [48] defines the calculation method for *R*^2^.

(22) $$\begin{array}{c} R^{2}=1-\frac{\sum_{i=1}^{n}{\left(y_{i}-y_{\bar{i}}\right)}^{2}/n}{\sum_{i=1}^{n}{\left(y_{i}-\bar{y}\right)}^{2}/n}\\ =1-\frac{MSE\left(\hat{y},y\right)}{\text{Var}\left(y\right)}, \end{array}$$

where the numerator in the rightest is the MSE, and the denominator is the variance of the actual value.

## 4. Results and Discussion

### 4.1. Results

#### 4.1.1. Model Processing

The dataset remains 2304296 instances with 53 features after preprocessing, feature selection, and feature encoding. This study builds the model using the Scikit-Learn ML toolkit on the Python platform with 8 cores and 16 GB RAM. To ensure reproducible results, all steps involving random processes set the random seed to 0.

The hyper-parameter *λ* in LR and RR models has the highest impact on performance. This study uses the default penalty coefficient *λ* = 1 in the toolkit. RFR, XGBR, and LightGBM are all tree-type models, and the hyper-parameter that most affects their performance is the number of CART regression trees (n_estimators). The more the number of trees, the higher the model performance may be, but the computing cost rises with it. The default n_estimators = 100 for RFR, and to facilitate the horizontal comparison of the three models, XGBR and LightGBM refer to the same order of magnitude of fitting time (Table 7) to set n_estimators to 500 and 25000, respectively. In particular, the LightGBM algorithm can set the number of features discarded ratio at each iteration to prevent overfitting, which is 0.6 in this study.

The article "Length of Stay Prediction Model of Indoor Patients Based on Light Gradient Boosting Machine" was published in 2022. Journal: Comput Intell Neurosci.

#### 4.1.2. Experimental Analysis

Table 7 shows the performance of models built with LR, RR, RFR, XGBR, and LightGBM algorithms, while the study results of Siddiqa et al. [16] are also listed side-by-side as a control. In the model of this study, the MSE (5.882) and *R*^2^ (0.675) metrics of LR on the test set are the worst, and its training time (3.654s) is also longer than another linear algorithm RR (1.653s). The performance of the RR algorithm (MSE = 5.680 and *R*^2^ = 0.702) outperforms the LR by a small margin, but the performance of both linear algorithms is far from satisfactory.

The RFR and XGBR-based models achieved MSE scores of 2.295 and 2.287, and the *R*^2^ scores are both 0.958 on the test set, which is well behaved as ideal. Their single-fold fitting consumption is 946.465s and 900.799s, respectively. However, the LightGBM algorithm surpasses them in fitting time (874.331s), MSE (2.231), and *R*^2^ (0.960), which performs best in the tree-type model.

Table 8 compares the performance variation of the best-performing LightGBM model in different encoding methods, where the hyper-parameter remains unchanged. In the results, label encoding (MSE = 2.248, *R*^2^ = 0.959), target encoding (MSE = 2.252, *R*^2^ = 0.959), and count encoding (MSE = 2.252, *R*^2^ = 0.959) have similar performance, while leave-one-out (MSE = 7.777, *R*^2^ = 0.221) performs the worst. And the proposed encoding (MSE = 2.231, *R*^2^ = 0.960) is the best method.

### 4.2. Discussion

The LR (*R*^2^ = 0.675) and RR (*R*^2^ = 0.702) models based on linear algorithms are far from ideal, which means that the datasets used in this study tend to be nonlinear, and linear algorithms are difficult to apply in practice to the process of predicting LOS. However, the three tree-type models (RFR, XGBR, and LightGBM) performed pretty well, especially the LightGBM model. Its *R*^2^ score of 0.960 is improved by 4.4% compared to the best-performing RFR model (5 MSE and 0.92 *R*^2^) in the past study [16] as the control group, while the MSE score of 2.231 is a relative decrease of 55.4%. XGBR and RFR models in this study ranked second and third in performance, with 2.5% and 2.8% respective higher MSE and 0.2% lower *R*^2^ scores relative to the best model.

Compared with the previous study [16], the encoding method in this study is a majority different. The models composed of LR, RR, RFR, and XGBR algorithms have significantly lower MSE scores (decreased by 86.3%, 85.2%, 54.1%, and 59.3% respectively) after using the proposed encoding method in this study, and *R*^2^ scores are improved (117.7%, 89.2%, 4.1%, and 5.5% higher). The LightGBM model using the proposed encoding also reduces the MSE score by at least 0.76% compared to label encoding, count encoding, target encoding, and leave-one-out encoding and *R*^2^ scores improved by at least 0.1%.

The article "Length of Stay Prediction Model of Indoor Patients Based on Light Gradient Boosting Machine" was published in 2022. Journal: Comput Intell Neurosci.

The model in this study can help the hospital to estimate the LOS of the patient, and the data to construct the model only need some prehospital diagnostic characteristics of the patient, thus reducing the threshold for the actual deployment and increasing the reality. In addition, the modeling process balances the conflict between the curse of dimensionality and information retention. Even for millions of instances, the model can be trained and deployed quickly using a personal computer. However, the model performance highly correlated with the “Total Charges” and “Total Costs” feature. Where “Total Charges” can be obtained when the patient admitted to the hospital, but “Total Costs” need to be estimated from the doctor's experience and other information about the patient. Uncertainty in the estimation results may affect model performance in reality.

## 5. Conclusions

The objective of this study was to construct a model to predict LOS in the hospital by exploring the prehospital diagnostic information of potential hospitalized patients. Many ML algorithms such as RFR, LR, RR, XGBR, MLP, and DTR are being investigated in recent studies for regression prediction of LOS. Eventually, the performance of the models constructed by these algorithms can hardly meet the requirements of actual deployment. Where the linear model is not suitable for predicting LOS and the tree model overfitting is obvious. This study proposed a model using one-hot encoding + label encoding combined with the LightGBM algorithm to investigate how to improve the accuracy of LOS prediction. The model is based on the 2017 dataset provided by the New York State Department of Health. The average LOS for patients in this dataset is 5.38 days, and most patients stay in the hospital for 1–5 days for minor illnesses, and more than 70% of illness types are medical. There was no significant difference in LOS between men and women, but over 50 spent more time in hospital. This study used a hybrid feature encoding approach to improve LOS prediction performance. And feature selection is also computed, which compared correlation scores to remove features that were not positive for prediction. The results of the correlation analysis showed that “Total Charges” and “Total Costs” were the features most associated with LOS. The proposed model ultimately successfully extends the results of related studies, with MSE and *R*^2^ achieving the best scores of 2.231 and 0.960, respectively, which is much higher than the previous study. In the future, the problem of model overfitting still deserves more research to obtain higher accuracy for predicting LOS.

The article "Length of Stay Prediction Model of Indoor Patients Based on Light Gradient Boosting Machine" was published in 2022. Journal: Comput Intell Neurosci.

## Figures and Tables

**Figure 1:** Visualization of the proposed framework.

**Figure 2:** Density plot of length of stay.

**Figure 3:** Length of stay distribution of two (three) class features.

**Figure 4:** Density plot of Total Costs and Total Charges.

**Figure 5:** Length of stay in Age Group and APR Risk of Mortality.

**Table 1:** Feature description of the dataset.

Feature name	Type	Description
Hospital Service Area	Radom categorical	Describe the location of the hospital
Hospital County		
Permanent Facility ID		Hospital service information
Facility Name		
Operating Certificate Number		Patient diagnostic information
Type of Admission		
CCS Diagnosis Code		
CCS Diagnosis Description		
CCS Procedure Code		
CCS Procedure Description		
APR DRG Code		
APR DRG Description		
APR MDC Code		
APR MDC Description		
APR Severity of Illness Code		
APR Severity of Illness Description		
Payment Typology 1		Patient cost information
Payment Typology 2		
Payment Typology 3		
Zip Code - 3 digits		Patient personal information
Race		
Ethnicity		
Patient Disposition		
Birth Weight		
Age Group	Ordered categorical	
APR Risk of Mortality		Patient diagnostic information
APR Medical Surgical Description	Three classes	
Gender		Patient personal information
Discharge Year	One class	Patient treatment information
Abortion Edit Indicator	Binary classes	
Emergency Department Indicator		Patient service information
Length of Stay	Continuous	Target feature
Total Charges		Patient cost information
Total Costs		

**Table 2:** Numerical conversion details of ordered categorical features.

Feature name	Original string data	Converted numerical data
Age Group	“0 to 17”	0
	“18 to 29”	1
	“30 to 49”	2
	“50 to 69”	3
	“70 or older”	4

APR Risk of Mortality	“Minor”	0
	“Moderate”	1
	“Major”	2
	“Extreme”	3

**Table 3:** Feature importance and selection results.

Feature name	Correlation or *P* value	Retain feature
Gender	0.053	Yes
APR Medical Surgical Description	0.043	
Emergency Department Indicator	0.051	
Hospital County	*P*=2.2*e* − 16	
Operating Certificate Number	*P*=2.2*e* − 16	
Permanent Facility Id	*P*=2.2*e* − 16	
Facility Name	*P*=2.2*e* − 16	
Zip Code - 3 digits	*P*=2.2*e* − 16	
CCS Diagnosis Code	*P*=2.2*e* − 16	
CCS Procedure Code	*P*=2.2*e* − 16	
APR DRG Code	*P*=2.2*e* − 16	
APR MDC Code	*P*=2.2*e* − 16	
Patient Disposition	*P*=2.2*e* − 16	
Hospital Service Area	*P*=2.2*e* − 16	
Ethnicity	*P*=2.2*e* − 16	
Type of Admission	*P*=2.2*e* − 16	
Payment Typology 1	*P*=2.2*e* − 16	
Race	*P*=2.2*e* − 16	
APR Severity of Illness Code	*P*=2.2*e* − 16	
APR Risk of Mortality	0.376	
Age Group	0.228	
Total Charges	0.602	
Total Costs	0.651	

The article "Length of Stay Prediction Model of Indoor Patients Based on Light Gradient Boosting Machine" was published in 2022. Journal: Comput Intell Neurosci.

**Table 4:** Label encoding example for the “Patient Disposition” feature.

Raw eigenvalues	Sorted eigenvalues	Numerical eigenvalues
Home or self-care	Short-term hospital	0
Skilled nursing home	Expired	1
Court/law enforcement	Hospice - medical facility	2
Skilled nursing home	Home or self-care	3
Court/law enforcement	Home or self-care	3
Short-term hospital	Skilled nursing home	4
Court/law enforcement	Skilled nursing home	4
Home or self-care	Court/law enforcement	5
Expired	Court/law enforcement	5
Hospice - medical facility	Court/law enforcement	5

**Table 5:** One-hot encoding example for the “Race” feature.

Raw feature	New features after numerical encoding		
Race	Race-White	Race-Black/African American	Race-other race
White	1	0	0
White	1	0	0
White	1	0	0
Black/African American	0	1	0
Black/African American	0	1	0
Black/African American	0	1	0
Black/African American	0	1	0
Other race	0	0	1
White	1	0	0

**Table 6:** The proposed encoding method.

Feature name	Encoding method
Gender	Label encoding
APR Medical Surgical Description	
Emergency Department Indicator	
Hospital County	
Operating Certificate Number	
Permanent Facility Id	
Facility Name	
Zip Code - 3 digits	
CCS Diagnosis Code	
CCS Procedure Code	
APR DRG Code	
APR MDC Code	
Patient Disposition	

Hospital Service Area	One-hot encoding
Ethnicity	
Type of Admission	
Payment Typology 1	
Race	
APR Severity of Illness Code	

APR Risk of Mortality	Sort the feature values from low to high and then encode them from 0 to N-1.
Age Group	

**Table 7:** Model performance in this and related study.

		Model performance in this study										
Model		LR			RR		RFR		XGBR		LightGBM	

MSE	Training	5.626			5.400		0.848		1.938		1.116	
	Test	5.882			5.680		2.295		2.287		2.231	

*R * ^2^	Training	0.697			0.726		0.994		0.969		0.990	
	Test	0.675			0.702		0.958		0.958		0.960	

Hyper-parameters		Alpha (*λ*) = 1			Alpha (*λ*) = 1		n_estimators = 100		n_estimators = 500		n_estimators = 25000 feature_fraction = 0.6	
One-fold fitting time		3.654s			1.653s		946.465		900.799s		874.331s	

Model performance in related study [16]												
Model			LR	RR		RFR		XGBR		MLP		DTR

MSE	Training		42.58	39		0.76		5.30		39		0.002
	Test		42.19	38.49		5		5.62		38.49		5.93

*R * ^2^	Training		0.31	0.37		0.987		0.914		0.37		0.999
	Test		0.31	0.3711		0.92		0.908		0.371		0.903

The article "Length of Stay Prediction Model of Indoor Patients Based on Light Gradient Boosting Machine" was published in 2022. Journal: Comput Intell Neurosci.

**Table 8:** The performance changes in different encoding methods.

Encoding Method	MSE		*R* ^2^	
	Training	Test	Training	Test
Label encoding	1.120	2.248	0.990	0.959
Count encoding	1.129	2.252	0.990	0.959
Target encoding	1.129	2.252	0.990	0.959
Leave-one-out encoding	0.023	7.777	0.999	0.221
Proposed encoding method	1.116	2.231	0.990	0.960

## Data Availability

The data that support the findings of this study are publicly available at https://health.data.ny.gov/Health/Hospital-Inpatient-Discharges-SPARCS-De-Identified/gaf8-ac33.
